# Investigating the Effects of EMGBF Combined with Different Motion Directions on Improving Upper Limb Function, iEMC, and Pain in Patients with Shoulder Dislocation

**DOI:** 10.1155/2023/1950150

**Published:** 2023-07-03

**Authors:** Di Wu, Jing Xu, Xiufang Lan

**Affiliations:** ^1^Department of Physical Education and Military, Zhejiang University of Technology, Hangzhou 310014, China; ^2^Traditional Chinese Medicine Rehabilitation, Hangzhou Massage Hospital (Hangzhou Minfu Hospital), Hangzhou 310009, China

## Abstract

The dislocation of the shoulder is a common complication of stroke, which is easy to occur after 3 months of stroke, with an incidence of 70%. There is no single standard for the pathogenesis of the disease, but the atrophy of the associated stability muscle, such as the triangle muscle, the oblique, and the upper muscle of the gonfield, may be the cause of the disease. In order to observe the effects of Electromyographic Biofeedback (EMGBF) combined with different motion directions on upper limb function with shoulder dislocation, a total of 84 patients with shoulder dislocation from May 2020 to February 2022 are selected for the study. The experimental results show that after treatment, upper limb motor function, iEMC, pain score, Barthel index, and quality of life score in the observation group are significantly higher than those in the control group, with statistical significance.

## 1. Introduction

Stroke has a high disability rate and high mortality rate and is prone to symptoms such as dizziness, nausea, and numbness of limbs, which seriously affect the physical function and daily life of patients [1]. Nowadays, the prevalence of this disease is gradually increasing, and the age of onset is gradually decreasing [2]. Shoulder dislocation is a common complication of stroke, which is easy to occur about 3 months after stroke, with an incidence of up to 70%. There is no unified standard for the pathogenesis of this disease, but paralysis and atrophy of the deltoid, trapezius, supraspinatus, and other related stable muscles may be the cause of this disease. After the onset of shoulder dislocation, the scapula and joint capsule are dislocated, breaking the original stable structure of the shoulder joint, resulting in the shoulder joint not being able to bear weight or support, and even unable to move normally.

If the treatment is not timely, the physical and mental health and quality of life of patients will be seriously affected. Therefore, it is extremely important to find scientific and effective methods to treat shoulder dislocation [3]. Electromyographic Biofeedback (EMGBF) is a new way of rehabilitation therapy, which takes the plasticity of the central nervous system as the entry point and provides feedback on exercise results through instruments [4]. EMGBF has significant efficacy in the treatment of neuromuscular diseases, which can provide a good basis for the clinical treatment of shoulder dislocation [5]. However, there are still some controversies in this method: the movement direction is single, the shoulder cannot be fully exercised, and there are limitations on the partial dislocation of the shoulder. Based on this, this study explores the effects of EMGBF combined with different motion directions in improving upper limb function, iEMC, and pain in patients with shoulder dislocation.

The rest of this paper is organized as follows: Section 2 discusses related work, followed by focusing on the general information and observation indicators in Section 3. The Fugl–Meyer upper limb motor function scores and VAS scores are discussed in Section 4.  Section 5 concludes the paper with summary.

## 2. Related Work

The shoulder joint was the highest and largest joint of the upper limb joint flexibility. The structure of the joint was that the joint capsule is thin and loose. There were muscles and tendons crossing on the upper, rear, and front of the joint capsule, but it lacked the strengthening of the anterior inferior muscle and tendon, so it was weak [6, 7]. In the analysis of anatomical and muscle mechanics abnormalities, it was found that stroke patients with hemiplegia would occur. The core part of the shoulder muscles in hemiplegia patients became loose, and the muscle tension of the shoulder joint would be lost, resulting in loss of control of the joint capsule and ligaments, and traction by gravity [8]. The clinical manifestations of this complication included shoulder pain, swelling, and disturbance in daily activities, etc. In severe cases, secondary axillary nerve injury would occur, thus affecting the normal motor function and quality of life of patients [9].

Generally, sling was the main method for treating shoulder dislocation, which could achieve good efficacy under static conditions, but frequent sitting and standing still aggravated the degree of dislocation [10]. Therefore, around 1965, EMGBF gradually emerged in the field of shoulder rehabilitation, widely used in the treatment of patients with physical disorders, patients could effectively feel their own behavior through the feedback of the instrument and could actively improve their own behavior to achieve the purpose of rehabilitation [11]. The upper limb motor function score of all patients after treatment was higher than before, and the upper limb function score of the observation group was higher than that of the control group after treatment (*P* < 0.05) [12]. The scholar found that after treatment, the upper limb function of patients in the extension group was significantly higher than that in the extension group and the abduction group, with statistical significance (*P* < 0.05). Mechanism analysis showed that patients with shoulder dislocation had low exercise awareness and poor compliance. EMGBF could make patients feel clear feedback after exercise. In the case of effectively improving the dislocation patient, the upper limb motor function of the patient could be further improved.

Some scholars have found that biofeedback therapy combined with point-to-line and surface acupuncture could effectively improve iEMC and quality of life score of patients [13]. VAS score and Barthel index in the observation group were significantly higher than those in the control group (*P* < 0.05) after the treatment of shoulder pain and the above results were consistent with the results of this study [14]. Barthel index, iEMC, pain score, and quality of life score of patients in the observation group were higher than those in the control group (*P* < 0.05). Analysis of its mechanism might be as follows: the core muscles of patients with shoulder dislocation were paralyzed, unable to resist the pressure of vertical gravity on the shoulder joint, resulting in impaired daily living ability and pain. The deltoid muscle was an important muscle group of the shoulder joint, which was headed by the acromion and tailed by the trochanter. Electromyographic biofeedback electrical stimulation therapy combined with the stimulation points of different movement directions was mainly in the deltoid muscle, which could exercise the deltoid muscle in all aspects and enhance the strength of the deltoid muscle bundle.

## 3. General Information and Observation Indicators

A total of 84 patients with shoulder dislocation treated in our hospital from May 2020 to February 2022 are selected as the study subjects and are divided into the observation group and control group according to random number table method. The observation group includes 42 patients, including 19 males and 23 females. The average age is 45.34 ± 8.31 years. There are 11 cases of dislocation of degree Ⅰ, 21 cases of dislocation of degree Ⅱ, and 10 cases of dislocation of degree Ⅲ. The control group includes 42 patients, including 22 males and 20 females. The average age is 44.58 ± 7.68 years. There are 10 cases of dislocation of degree Ⅰ, 20 cases of dislocation of degree Ⅱ, and 12 cases of dislocation of degree Ⅲ. There is no significant difference in general data between the two groups (*P* > 0.05). Patients who are involuntary and unable to communicate are excluded.

The control group receives conventional drugs and rehabilitation treatment and EMGBF treatment is added on this basis. The observation group is supplemented with EMGBF treatment in different motion directions on the basis of the control group. The specific contents are as follows: The medical staff will introduce the treatment methods, effects, and precautions to the patients and their families before treatment, reduce the psychological pressure on the patients and their families, and strengthen the cooperation of the patients and their families. The biological stimulation feedback instrument (SA9800) of Canada Thought Teach is used for the EMGBF instrument. The patient sits in front of the monitor, and the treatment position of the patient's electrode is sterilized with 75% ethanol and firmly affixed with the electrode. The position of the electrode is divided into three kinds according to the direction of movement: (1) Forward flexion exercise: in the anterior deltoid muscle bundle, the patient does shoulder flexion exercise as required. (2) Posterior extension exercise: in the posterior deltoid muscle bundle, the patient does shoulder extension exercises as required. (3) Abduction exercise: in the middle bundle of deltoid muscle, the patient performs shoulder abduction exercises as required. Before the patient moves, the medical staff should demonstrate the normal movement, and let the patient feel the electrical stimulation in advance to avoid panic, and at the same time, the patient can remember this feeling in advance. The EMG signal on the monitor can show muscle strength, which requires careful observation by the patient. The patient needs to operate under the joint command of the instrument and the doctor. The instrument command is “refueling”. When the doctor gives a force command, the patient will do as much standard action as possible under the command, the patient's output reaches the critical value, and the patient will receive electrical stimulation feedback from the instrument. The instrument indicates “maintenance”. When the doctor gives maintenance instructions, the patient needs to keep the muscles contracted at an isometric distance and keep moving. The command is “relax”. When the doctor gives the rest command, the patient needs to completely relax the target muscle. The course of treatment is 25 min/time, 4 times/week for 8 weeks.

Observation indicators are as follows: (1) the Fugl–Meyer is used to assess the motor function of the upper limbs. (2) iEMC scores of patients in the two groups at different times are observed, and the 10-channel surface dynamic tester is used. The higher the score, the better the muscle strength. (3) VAS score is used to evaluate the pain degree. (4) Barthel index of two groups before and after treatment is observed. (5) Stroke Specific Quality of Life Scale (SSQOLS) is used to evaluate the quality of life. The higher the score, the better the quality of life of patients.

In this study, all the data and the corresponding database are established. All data processing is entered into SPSS 26.0, including the normal test of measurement data, expressed as (*x* + *s*). Repeated measures analysis of variance and spherical line test are used. *P* < 0.05, the difference is statistically significant.

## 4. Fugl–Meyer Upper Limb Motor Function Scores and VAS Scores

### 4.1. Fugl–Meyer Upper Limb Motor Function Scores

Table 1 is the comparison of Fugl–Meyer upper limb motor function scores before and after treatment between the two groups. It is clearly evident from Table 1 that the upper limb function score of two groups after treatment is significantly higher than that before treatment, and the upper limb function score of the observation group is significantly higher than that of the control group after treatment (*P* < 0.05).

### 4.2. iEMC Scores of the Two Groups

Table 2 is the comparison of iEMC scores. It is clearly evident from Table 2 that the iEMC scores of the two groups after treatment are significantly higher than those before treatment.

Figure 1 is the comparison of iEMC scores. It is clearly evident from Figure 1 that iEMC scores of the observation group at 3, 6, and 8 weeks after treatment are higher than those of the control group (*P* < 0.05).

### 4.3. VAS Scores of the Two Groups

Table 3 is the comparison of pain VAS scores. It is clearly evident from Table 3 that the pain in both groups is significantly reduced after treatment, and the pain score in the observation group is significantly lower than that in the control group (*P* < 0.05).

### 4.4. Barthel Index of the Two Groups

Table 4 is the comparison of Barthel index. It is clearly evident from Table 4 that the Barthel index of the observation group is significantly higher than that of the control group after treatment (*P* < 0.05).

### 4.5. Quality of Life Scores of the Two Groups

Table 5 is the comparison of the quality of life scores. It is clearly evident from Table 5 that the score of quality of life after treatment is higher in both groups than before, and the score of quality of life after treatment in the observation group is significantly higher than that in the control group (*P* < 0.05).

## 5. Conclusion

The shoulder joint is the highest and largest joint of the upper limb joint flexibility. Therefore, common shoulder articulation is usually caused by anterior and lower shoulder articulation. In this paper, a total of 84 patients with shoulder dislocation from May 2020 to February 2022 are selected to observe the effects of EMGBF combined with different motion directions on upper limb function. The experimental results show that EMGBF combined with different motion direction therapy can effectively improve the iEMC of patients with shoulder dislocation, and can enhance the upper limb motor function and daily living ability of patients, relieve pain of patients, so as to further improve patients' quality of life, increase patients' confidence in treatment, and reduce patients' stress. However, due to the small sample size of this study, it is not highly representative. Further studies on the sample size and molecular mechanism can be carried out to further demonstrate the changes of indicators in this study.

## Figures and Tables

**Figure 1:** Comparison of iEMC scores.

**Table 1:** Comparison of Fugl–Meyer upper limb motor function scores before and after treatment between the two groups (*x ± s*, score).

Group	Number	Fugl–Meyer upper limb motor function scores		*t*	*P*-value
		Before treatment	After treatment		
Observation group	42	24.37 ± 7.61	49.86 ± 10.22	5.331	0.001
Control group	42	25.19 ± 7.42	40.11 ± 4.31	4.236	0.001
*t*		4.334	5.526		
*P*		0.001	0.001		

**Table 2:** Comparison of iEMC scores (*x ± s*, score).

Group	Time	iEMC
Observation group (*n* = 42)	Before treatment	0.64 ± 0.06
	3 weeks after treatment	0.67 ± 0.07
	6 weeks after treatment	0.74 ± 0.06
	8 weeks after treatment	0.79 ± 0.07

Control group (*n* = 42)	Before treatment	0.63 ± 0.05
	3 weeks after treatment	0.65 ± 0.06
	6 weeks after treatment	0.66 ± 0.06
	8 weeks after treatment	0.67 ± 0.07

*F*_time_		9.371
*P*_time_		<0.001
*F*_time_ *×* group		9.887
*P*_time_ *×* group		<0.001

**Table 3:** Comparison of pain VAS scores (*x ± s*, score).

Group	Number	VAS		*t*	*P*-value
		Before treatment	After treatment		
Observation group	42	4.37 ± 1.02	1.07 ± 0.03	6.423	0.001
Control group	42	4.09 ± 1.35	2.79 ± 0.06	5.321	0.001
*t*		6.547	4.374		
*P*		0.001	0.001		

**Table 4:** Comparison of Barthel index (*x ± s*, score).

Group	Number	Barthel index		*t*	*P*-value
		Before treatment	After treatment		
Observation group	42	18.24 ± 6.09	47.33 ± 9.54	5.342	0.001
Control group	42	19.21 ± 5.27	38.76 ± 9.01	5.078	0.001
*t*		5.754	5.343		
*P*		0.001	0.001		

**Table 5:** Comparison of the quality of life scores (*x ± s*, score).

Group	Number	Quality of life scores		*t*	*P*-value
		Before treatment	After treatment		
Observation group	42	114.31 ± 37.69	146.82 ± 40.09	7.214	0.001
Control group	42	116.57 ± 36.97	137.48 ± 36.98	6.156	0.001
*t*		7.478	6.543		
*P*		0.001	0.001		

## Data Availability

The simulation experiment data used to support the findings of this study are available from the corresponding author upon request.
